# Analysis of the Effectiveness of SMILE, FS-LASIK, and SBK in Myopic Patients and the Impact in UCVA and Tear Film Stability

**DOI:** 10.1155/2022/6233232

**Published:** 2022-07-31

**Authors:** Yan Ji, Wenjuan Wan, Qi Zhang, Mei Xu, Xin Yang, Jiuyi Xia

**Affiliations:** Department of Ophtalmology, The First Affiliated Hospital of Chongqing Medical University, Chongqing Key Laboratory of Ophthalmology and Chongqing Eye Institute, Chongqing 400000, China

## Abstract

The aim of the present study was to investigate the effect of femtosecond laser small incision stromal lens extraction (SMILE), femtosecond laser-assisted excimer laser keratomileusis (FS-LASIK), and anterior elastic sublaminar laser keratomileusis (SBK) in myopic patients, and their effects on uncorrected visual acuity (UCVA) and tear film stability. 600 myopic patients admitted to our hospital from January 2020 to December 2021 were selected for the study and divided into SMILE group (200 patients, SMILE treatment), FS-LASIK group (200 patients, FS-LASIK treatment), and SBK group (200 patients, SBK treatment) according to the random number table method. Uncorrected visual acuity (UCVA), tear breakup time (BUT), tear secretion function test (Sit), and corneal higher-order image aberration global higher-order aberration (HOAS) were compared among the three groups. The UCVA values before operation, 2 weeks after operation, 1 month after operation, and 3 months after operation in the three groups were similar, and the BUT, Sit value, and HOAS of corneal higher-order image difference in the three groups were similar, and the differences were not statistically significant (*P* > 0.05). The BUT, Sit value, and HOAS of corneal higher-order image difference at 1 and 3 months after surgery in the SMILE group were higher than those in the FS-LASIK and SBK groups, and the differences were statistically significant (*P* < 0.05). SMILE, FS-LASIK, and SBK are effective in the treatment of myopia, which can effectively improve the uncorrected visual acuity and help the patients to recover their normal visual ability, but SMILE is more effective in tear film stability and corneal higher-order aberrations.

## 1. Introduction

Myopia is a type of refractive error in which parallel light enters the eye (when the eye is relaxed) and is focused in front of the retina, causing blurring of the image on the retina and inducing typical symptoms such as visual fatigue and loss of distance vision. As myopia increases, it can be accompanied by symptoms such as obscuration, distortion, and double vision, which can aggravate the damage to the fundus of the eye and cause irreversible damage to the patient's vision [1, 2]. With the development of medical technology, myopia correction surgery is more and more widely used, and the surgical methods are also more and more diverse [3]. Due to individual differences, there are some differences in the actual efficacy of various myopia correction surgeries, of which femtosecond laser small incision lenticule extraction (SMILE) has the advantages of small incision, no need for corneal flap creation and fast recovery after surgery [4]. Femtosecond laser in situ keratomileusis (FS-LASIK) is one of the mainstream corneal refractive surgeries with the advantages of precise flap creation, convenience, and rapid recovery [5]. Sub-Bowmans Keratomileusis (SBK) is a novel LASIK procedure that can create ultrathin flaps of 90–100 *μ*m thickness (containing Descemet's membrane and a little underlying stroma) with the advantages of a wide range of use and stable results [6]. Therefore, this study intends to conduct a comparative study on the practical effects of SMILE, FS-LASIK, and SBK in myopia. The effects of these three procedures on patients' visual ability and ocular structural function will be further explored to provide a reference for myopia surgical treatment.

## 2. Patients and Methods

### 2.1. Patients

From January 2020 to December 2021, 600 myopic patients were selected and admitted to our hospital. The diagnostic criteria were as follows: all patients met the diagnostic criteria for myopia [7]. The inclusion criteria were as follows:

1. Patients all aged 18–40 years old;
2. All had symptoms of asthenopia and distance vision loss;
3. Basic information is complete;
4. Patients with myopia < −10.00D, astigmatism < −6.00D, corneal curvature 40–46D, and pupil diameter within 6 mm;
5. Patients and their families voluntarily signed informed consent.

The exclusion criteria were as follows:

1. Cornea was too thin to meet the surgical criteria;
2. There were eyelid defects, deformation, and other serious ocular structural lesions;
3. There were other serious ophthalmic diseases, such as cataracts and glaucoma;
4. There were autoimmune diseases;
5. There were serious infectious diseases before this study;
6. There were mental illnesses, language barriers, and too low cooperation.

According to the random number table, they were divided into the SMILE group (200 cases, SMILE treatment), FS-LASIK group (200 cases, FS-LASIK treatment), and SBK group (200 cases, SBK treatment). There was no significant difference in the basic data (age, surgical eye, intraocular pressure, and gender composition) between the two groups (*P* > 0.05) (Table 1). The research program is fully in line with the Helsinki Declaration. It was approved by The First Affiliated Hospital of Chongqing Medical University's Medical Ethics Committee.

### 2.2. Methods

In the SMILE group, SMILE treatment was implemented. The patient was placed in the supine position, surface anesthesia was administered with 4 g/L oxybuprocaine hydrochloride eye drops (Shiga Plant, Santen Pharmaceutical Co. Ltd., Japan, Spec. 20 ml: 80 mg/box) and the lids were opened with a lid opener (Kang Hong, ciliary masking). With a full femtosecond laser refractive surgery system (VisuMax, CarlZeiss, Germany), the eye was centrally positioned with microscopic support, fixed by negative pressure suction, and the device parameters were adjusted to a laser energy of 500 kHz and 130 nJ, a side cutting angle of 90°, a width of 2 mm, a lens diameter of 6.0–6.5 mm, and a design corneal flap thickness of 120–130 *μ*m. After prescanning (the corneal interlayer), the corneal stromal lens was cut and prepared, the stromal lens was removed (a microincision is made to separate the stromal lens for removal), and the corneal stromal bed was rinsed with equilibration solution.

In the FS-LASIK group, FS-LASIK treatment was performed. FS-LASIK treatment was performed. The patient was placed in the supine position, surface anesthesia was administered with 4 g/L oxybuprocaine hydrochloride drops, and the lid was opened with a lid opener. A corneal flap was created using a full femtosecond laser refractive surgery system with parameters set at 185 nJ laser energy, 90–110 *μ*m flap thickness, 7.9–8.5 mm flap diameter, 4.10 mm flap width, and a tip located above the cornea. Corneal stromal cutting (LASIK cutting method, 250 kHz laser) was then completed with an excimer laser (VISXSTARs4, Nuctech, USA). This was followed by flushing (balanced salt solution), resetting the flap, drying, and wrapping the eye (rigid eye shield).

In the SBK group, SBK treatment was performed. In the supine position, surface anesthesia was administered with 4 g/L oxybuprocaine hydrochloride drops and the lid was opened with a lid opener. A corneal flap (tip in the nasal cornea, diameter 8.0 mm) was created with a corneal lamellar knife (Moria One Use-Plus (90 *μ*m), France), the flap was lifted and cut with an excimer laser in a small spot pattern (light zone diameter 6.0 mm), the stromal bed was flushed and the flap is repositioned.

All three study groups received regular postoperative medication, including tobramycin dexamethasone eye drops (Hangzhou Guoguang Pharmaceutical Co. Ltd., State Pharmacopoeia H20073641, Specification 5 ml: 15 mg: 5 mg/box), 4 times/d, 1–2 drops/time, for 7 d; and sodium vitrate eye drops (URSAPHARM Arzneimittel GmbH, Germany. Registration No. H20150150, size 0.1% (preservative-free) 10 ml/box), 4 times/d, 1–2 drops/dose, for 2 months of treatment.

### 2.3. Observation Indicators

Uncorrected visual acuity (UCVA) was compared among the three groups: before surgery and at 2 weeks, 1 month, and 3 months after surgery, the patients were tested for uncorrected visual acuity (without frame glasses, contact lenses, etc.) with a visual acuity chart according to the relevant standards, and uncorrected visual acuity ≥1.0 in one eye was considered normal. The mean UCVA value of the patient's surgical eye was counted.

Endometrial stability was compared among the three groups: tear breakup time (BUT) and tear secretion function test (Schirmer I test, Sit) were performed preoperatively, at 1 month and 3 months. The BUT was to place the standard fluorescein filter paper at the lower palpebral conjunctival sac, we instructed the patient to blink 3–5 times and then take it out, we observed under the illumination of a slit lamp drill blue lamp, counted the time from the last blink to the occurrence of a dry spot on the tear film, and detected the mean value for 3 times at each time period. After Sit detected the reflected end of the filter paper strip (5 mm) with tears, it was placed at the lower eyelid margin and the patient was allowed to close his eyes lightly and removed 5 minutes later to record the degree of filter paper wetness.

Corneal high-order aberrations (HOASs) were compared among the three groups: HOAS was measured with a wavefront aberration analyzer (OPD-SCAN) before surgery and at 1 and 3 months after surgery, and the mean value was measured twice.

### 2.4. Statistical Analysis

Statistical Product and Service Solutions (SPSS) 23.0 (IBM, Armonk, NY, USA) was applied for statistical analysis. An independent sample *t*-test was used for comparison between groups for measurement data obeying normal distribution, and an independent sample *t*-test was used for comparison within groups, all expressed as ($\bar{x}$ ± *s*). Count data were tested by *χ*2 and expressed as rate (%), and *P* < 0.05 indicates a statistical difference.

## 3. Results

### 3.1. UCVA in the Three Groups

The UCVA values of the three groups were similar before surgery, 2 weeks after surgery, 1 month after surgery, and 3 months after surgery, and the difference was not statistically significant (*P* > 0.05) (Table 2).

### 3.2. Intimal Stability among the Three Groups

The BUT and Sit values of the three groups were similar, and the difference was not statistically significant (*P* > 0.05). The BUT and Sit in the SMILE group were higher than those in the FS-LASIK and SBK groups at 1 and 3 months after surgery, and the differences were statistically significant (*P* < 0.05) (Table 3).

### 3.3. The Corneal Higher Order Image Difference HOAS of the Three Groups

The corneal higher-order image difference HOAS of the three groups was similar, and the difference was not statistically significant (*P* > 0.05). The corneal higher-order image difference HOAS at 1 and 3 months after surgery in the SMILE group was higher than that in the FS-LASIK and SBK groups, and the difference was statistically significant (*P* < 0.05) (Table 4).

## 4. Discussion

Myopia is a common eye disease today. The exact cause of myopia is not known, but numerous studies have shown that myopia has a genetic predisposition, while environmental factors, such as long reading hours, poor lighting and lack of outdoor activities, can increase the risk of myopia [8, 9]. In addition, studies have found that micronutrient deficiencies, nutrient imbalances and prolonged close viewing of electronic devices are all common triggers of myopia, so those with these risk factors and triggers need to pay attention to the prevention and treatment of myopia [9].

Frame eye is a common treatment for myopia. The effective wearing of frame glasses can relieve asthenopia and improve visual ability by correcting visual acuity. However, the effect of conventional frame eye and drug treatment is limited, and the purpose of radical treatment cannot be achieved. Myopia correction surgery such as corneal refractive surgery and intraocular lens implantation has a certain curative effect. In recent years, the number of myopic patients receiving surgical treatment is also increasing. According to the patient's condition, diagnosis and treatment budget, existing surgical equipment, etc., providing the most appropriate surgical method for patients has a positive impact on promoting the establishment of a good doctor-patient relationship and improving the efficacy of surgery.

In this study, SMILE, FS-LASIK, and SBK were compared and analyzed in depth. The results showed that the UCVA values of the three groups before surgery, 2 weeks after surgery, 1 month after surgery and 3 months after surgery were similar (*P* > 0.05), suggesting that these three surgical treatment methods could effectively improve the incorrected visual acuity of myopic patients and improve the symptoms of distance vision loss. The reasons for this may be as follows: all three procedures, SMILE, FS-LASIK, and SBK, were corneal refractive surgeries based on laser technology, and with laser technical support, these three procedures had the advantages of short treatment time (the required pulse can be obtained in a very short time), small focusing space, high accuracy, and little damage to surrounding tissues and organs [10]. The cornea has the effect of providing most of the refractive power for the eye. Combined with the refractive power of the lens, the parallel light can be focused on the retina and form a clear image after entering the eye [11].

Corneal refractive surgery helps myopic patients recover more normal corneal refractive power by adjusting the corneal thickness, shape, etc., in order to improve the visual ability of myopic patients and help patients restore normal vision [12]. In terms of surgical efficacy, this study showed that the BUT, Sit value, and corneal higher-order image difference HOAS at 1 and 3 months after surgery in the SMILE group were higher than those in the FS-LASIK and SBK groups (*P* < 0.05), suggesting that SMILE was beneficial to improve tear film stability and improved the effect of surgical treatment on corneal higher-order aberrations. This may be due to the fact that SMILE does not require the creation of a flap, but only a laser to create a corneal stromal lens, which is a more closed procedure and can further reduce the damage to the tissues and nerves of the eye from the surgical treatment [13].

Corneal flaps need to be made in both FS-LASIK and SBK. During laser ablation, it is easy to damage the afferent sensory nerve fibers promoted by the cornea, resulting in the destruction of the nerve reflex arc at this site, affecting the eye closure guided by nerve conduction, secretion of tears and other movements, resulting in a decrease in the frequency of eye closure and tear secretion after surgery and inducing dry eye symptoms. At the same time, compared with FS-LASIK and SBK, SMILE caused less surgical trauma, could protect the biomechanical properties of the cornea to the greatest extent, effectively avoided aberration changes due to the flap, and further improved the recovery effect of the patient's postoperative visual ability. Studies [14] found that the improvement of corneal aberration was superior in myopic patients treated with SMILE, which was consistent with the results of this study. This study is a single-centre study with a small sample size, so the conclusions drawn still need to be further confirmed by a multicentre, randomised, double-blind, large sample study.

## 5. Conclusion

In summary, SMILE, FS-LASIK, and SBK have ideal surgical results in myopia, which can effectively improve the uncorrected visual acuity of patients and help patients recover more normal visual ability, but SMILE has a better effect on tear film stability and corneal higher-order aberrations.

## Figures and Tables

**Table 1:** Comparison of basic data (x̅ ± *s*, n).

Group	Number of subjects	Age (years)		Operative eye		Intraocular pressure (mmHg)		Gender composition	
		Scope	Average	Scope	Average	Scope	Average	Male	Female
SMILE group	200	18–39	28.59 ± 4.12	361–400	380.52 ± 8.23	10–21	15.52 ± 4.12	101 (50.50%)	99 (49.50%)
FS-LASIK group	200	18–40	29.01 ± 4.56	358–400	379.04 ± 8.01	11–19	15.04 ± 4.03	106 (53.00%)	94 (47.00%)
SBK group	200	21–38	29.51 ± 4.96	359–399	379.07 ± 8.18	11–21	16.04 ± 4.75	89 (44.50%)	111 (55.50%)
Χ^2^/F	-	2.040		2.160		2.690		3.054	
*P* value	-	0.131		0.116		0.069		1.217	

**Table 2:** Comparison of the UCVA of the three groups (x̅ ± *s*, LogMAR).

Group	Number of subjects	Pre-op	2 weeks after surgery	1 month post-op	3 months after operation
SMILE group	200	0.57 ± 0.12	0.91 ± 0.22	1.01 ± 0.24	1.03 ± 0.25
FS-LASIK group	200	0.58 ± 0.14	0.95 ± 0.25	1.02 ± 0.22	1.01 ± 0.23
SBK group	200	0.56 ± 0.17	0.93 ± 0.24	1.00 ± 0.23	1.01 ± 0.25
F	-	0.950	1.420	0.380	0.450
*P* value	-	0.386	0.242	0.686	0.638

**Table 3:** Compares the intimal stability of the three groups (x̅ ± *s*).

Group	Number of subjects	BUT (s)			Sit (mm/5 min)		
		Pre-op	1 month post-op	3 months after operation	Pre-op	1 month post-op	3 months after operation
SMILE group	200	9.14 ± 2.11	5.23 ± 1.21	7.27 ± 1.86	14.97 ± 3.12	9.32 ± 2.15	12.71 ± 3.02
FS-LASIK group	200	9.17 ± 2.14	4.86 ± 1.25	5.56 ± 1.28	15.01 ± 3.54	8.86 ± 2.01	10.04 ± 2.93
SBK group	200	9.11 ± 2.10	4.91 ± 1.22	5.92 ± 1.54	14.96 ± 3.34	8.89 ± 2.05	9.89 ± 2.85
F	-	0.040	5.360	65.280	0.010	3.030	58.480
*P* value	-	0.961	0.005	0.001	0.988	0.049	0.001

**Table 4:** Comparison of the corneal higher-order image difference HOAS of the three groups [x̅ ± *s*].

Group	Number of subjects	Pre-op	1 month post-op	3 months after operation
SMILE group	200	0.28 ± 0.08	0.96 ± 0.11	0.97 ± 0.14
FS-LASIK group	200	0.27 ± 0.06	0.48 ± 0.84	0.47 ± 0.10
SBK group	200	0.28 ± 0.07	0.59 ± 0.95	0.61 ± 0.98
F	-	1.340	23.420	40.320
*P* value	-	0.262	0.001	1.1

## Data Availability

The datasets used and analyzed during the current study are available from the corresponding author on reasonable request.
